# Markers of Inflammation, Oxidative Stress, and Fibrosis in Patients with Atrial Fibrillation

**DOI:** 10.1155/2022/4556671

**Published:** 2022-05-23

**Authors:** Priit Pauklin, Mihkel Zilmer, Jaan Eha, Kaspar Tootsi, Mart Kals, Priit Kampus

**Affiliations:** ^1^Department of Cardiology, Institute of Clinical Medicine, University of Tartu, 8 Puusepa Street, Tartu 51014, Estonia; ^2^Heart Clinic, Tartu University Hospital, 8 Puusepa Street, Tartu 51014, Estonia; ^3^Department of Biochemistry, Institute of Biomedicine and Translational Medicine, Centre of Excellence for Genomics and Translational Medicine, University of Tartu, 19 Ravila Street, Tartu 50411, Estonia; ^4^Department of Traumatology and Orthopedics, Institute of Clinical Medicine, University of Tartu, 8 Puusepa Street, Tartu 51014, Estonia; ^5^Estonian Genome Center, Institute of Genomics, University of Tartu, 23b Riia Street, Tartu 51010, Estonia; ^6^Institute for Molecular Medicine Finland, FIMM, HiLIFE, University of Helsinki, 8 Tukholmankatu Street, Helsinki 00290, Finland; ^7^Centre of Cardiology, North Estonia Medical Centre, 19 Sütiste Street, Tallinn 13419, Estonia

## Abstract

Atrial fibrillation (AF) is the most common sustained cardiac arrhythmia in clinical practice. The pathogenesis of AF is linked to inflammatory reaction and oxidative stress, which leads to fibrosis of the atria and progression of the disease. The purpose of this study was to define the role of several biomarkers of inflammation, fibrosis, and oxidative stress (OxS). We included 75 patients with paroxysmal/persistent AF, who were admitted for electrical cardioversion or pulmonary vein isolation (PVI). High-sensitivity C-reactive protein (hsCRP), galectin-3 (Gal-3), myeloperoxidase (MPO), oxidized low-density lipoprotein (oxLDL), and N-terminal pro-brain natriuretic peptide (NT-proBNP) were measured before the procedures. We compared the results with those of 75 healthy age-, sex-, and blood pressure-matched individuals. The patients were followed up for 1 year after the intervention to establish the recurrence of AF and its association with the measured markers. Patients with AF had higher MPO (52.6 vs. 36.2 ng/ml, *p* < 0.001) and NT-proBNP (209.0 vs. 28.0 pg/ml, *p* < 0.001) compared to healthy subjects. Also, they showed significantly higher levels of hsCRP (1.5 vs. 1.1 mg/l, *p* = 0.001) and Gal-3 (11.4 vs. 9.7 mg/l, *p* = 0.003), while there was no difference found in oxLDL (71.5 vs. 71.7 U/l, *p* = 0.449). MPO (OR = 1.012, *p* = 0.014), hsCRP (OR = 1.265, *p* = 0.026), and weight (OR = 1.029, *p* = 0.013) were independently associated with AF in a multivariable logistic regression analysis. Patients with successful maintenance of sinus rhythm (SR) for one year had lower baseline MPO (40.5 vs. 84.3 ng/ml, *p* = 0.005) and NT-proBNP (127.5 vs. 694.0 pg/ml, *p* < 0.001) compared to patients with recurrent AF episodes, but there was no difference in hsCRP, Gal-3, or oxLDL between them. MPO (OR = 0.985, *p* = 0.010) was independently associated with AF recurrence during the follow-up period when adjusted for cofounders. Patients with AF had increased markers of inflammation and fibrosis, while there was no increase detected in the OxS marker oxLDL. MPO was independently associated with AF in a multivariate model. Inflammatory and fibrotic mechanisms are important factors in electrical and structural remodelling progress in the atria of patients with AF.

## 1. Introduction

Atrial fibrillation (AF) is the most common sustained cardiac arrhythmia and is frequently encountered in everyday clinical practice. The development of AF is complex and is outlined by changes in the electrical and mechanical properties of the atria [1].

The association of cardiovascular disease with low-grade inflammation has been documented in multiple cases. Studies have confirmed the link to hypertension, coronary artery disease, and also obesity [2–4]. In recent years, an increasing number of studies have shown the importance of inflammation in the pathophysiological mechanisms that may lead to left atrial fibrosis and AF [5, 6].

Data on pathways involving processes of oxidative stress (OxS) also suggest their contribution to atrial remodelling and development of AF [7–10].

However, the importance of OxS versus inflammation and their interactions are not clearly established in patients with AF. Also, only a few studies have examined the prognostic importance of biomarkers in maintaining sinus rhythm (SR) in patients with AF who are managed with rhythm control therapy. The purpose of this study was to define the role of several biomarkers of inflammation (high-sensitivity C-reactive protein (hsCRP), galectin-3 (Gal-3)), OxS (oxidized low-density lipoprotein (oxLDL)), and fibrosis (myeloperoxidase (MPO), N-terminal pro-brain natriuretic peptide (NT-proBNP)) in patients with AF episodes. Our secondary goal was to assess their predictive value in maintaining SR.

## 2. Methods

### 2.1. Study Population

We included 75 patients with paroxysmal/persistent AF hospitalized for aggressive rhythm control therapy (electrical cardioversion or pulmonary vein isolation (PVI)) to the Department of Cardiology, Tartu University Hospital, and to the Centre of Cardiology, North Estonia Medical Centre, Estonia, respectively. We included patients between 18 and 75 years and only with successful electrical cardioversion to SR or SR before PVI procedure [11, 12]. Patients with failure to cardiovert to SR were excluded. Patients with heart failure, valve pathology (moderate to severe), known inflammatory disease, or history of cancer were also excluded. We used age-, sex-, and blood pressure- (BP-) matched subjects without a history of any arrhythmias as a control group. These subjects were recruited from general practitioners' practices. As with the study group, individuals with a history of heart failure, valve pathologies, cancer, or inflammatory disease were excluded. The study was approved by the Research Ethics Committee of the University of Tartu and was conducted in accordance with the Declaration of Helsinki. Each participant signed a written consent before the study.

### 2.2. Study Protocol

Venous blood samples were collected after an overnight fast, but before electrical cardioversion or PVI. Blood pressure (BP) was measured after 15 minutes of rest in a quiet, temperature-controlled special study room in a supine position. Patients were followed up for 1 year after either electrical cardioversion or PVI to assess recurrence of AF.

### 2.3. Hemodynamic Measurements

For BP measurements, a validated digital oscillometric device (A&D UA-767; A&D Company Ltd., Tokyo, Japan) was used at least twice and mean BP was used in the study.

### 2.4. Laboratory Analysis

hsCRP and NT-proBNP were measured with commercially available assays, using standard laboratory methods, at the local clinical laboratory. Gal-3 was measured using the ARCHITECT galectin-3 assay kit, employing chemiluminescent microparticle immunoassay (CMIA) technology. MPO was measured using the BIOCHECK myeloperoxidase enzyme immunoassay kit, and oxLDL was measured using the MERCODIA oxidized LDL kit, both by employing the enzyme-linked immunosorbent assay (ELISA) technology.

### 2.5. Follow-Up

Patients were monitored using ECG telemetry for at least one day after successful electrical cardioversion or PVI at the hospital. After discharge, patients were monitored for AF recurrence at 3-4 months, 6 months, and 1 year after electrical cardioversion. Standard 12-lead ECGs were obtained at each visit, and patients were questioned about rhythm disturbances. Holter monitoring was done 3 months after PVI. Electronic medical records were followed up for one year after the procedures, regarding documented rhythm disturbances. The endpoint was documentation of new AF episodes during follow-up.

The control group was also followed up, remotely, for the same period. Electronic medical records, ECGs, and family physician's electronic notes were checked for the diagnosis of AF.

Successful maintenance of SR was defined as the absence of documented AF on ECG, or 24-hour Holter monitor during the 1-year follow-up period, or absence of medical contact because of rhythm disturbances.

### 2.6. Statistical Analysis

Continuous variables were summarized using mean ± standard deviations (SD), and statistical differences between groups were tested using Student's *t*-test. Alternatively, median with interquartile range (IQR) was used to characterize biomarkers with nonparametric Mann–Whitney *U* test for group comparison. Categorical variables were presented as counts with proportions (%) and tested by the chi-squared test.

To identify independent risk factors for the association of AF, all variables of univariate analyses with *p* value < 0.15 were included in the multivariable logistic regression model and backward elimination was used for variable selection. A *p* value of <0.05 was considered statistically significant. All statistical analyses were performed using R [13], version 3.6.3.

## 3. Results

### 3.1. Laboratory Measurements

Patients with AF had higher MPO (52.6 vs. 36.2 ng/ml, *p* < 0.001) and NT-proBNP (209.0 vs. 28.0 pg/ml, *p* < 0.001) compared to healthy subjects. Also, they had significantly higher hsCRP (1.5 vs. 1.1 mg/l, *p* = 0.001) and Gal-3 (11.4 vs. 9.7 mg/l, *p* = 0.003). There was no difference in oxLDL levels (71.5 vs. 71.7 U/l, *p* = 0.449) between AF patients and controls (Table 1, Figure 1). Multivariable logistic regression analysis showed that MPO (OR = 1.012, *p* = 0.014), hsCRP (OR = 1.265, *p* = 0.026), and weight (OR = 1.029, *p* = 0.013) were independently associated with AF (Table 2).

### 3.2. Follow-Up

During the follow-up period of the study group, 30 patients had AF recurrence.

Baseline MPO was lower in the SR subgroup compared to those who had recurrent episodes of AF during one-year follow-up (40.5 vs. 84.3 ng/ml, *p* = 0.005). Lower NT-proBNP values were observed in the SR subgroup (127.5 vs. 694.0 pg/ml, *p* < 0.001). At the same time, there were no statistically significant differences detected in hsCRP (1.5 vs. 1.9 mg/l, *p* = 0.859), Gal-3 (10.8 vs. 11.8 mg/l, *p* = 0.355), or oxLDL (75.7 vs. 67.2 U/l, *p* = 0.107) (Figure 2).

The characteristics of patients with successful and unsuccessful maintenance of SR are shown in Table 3. The table also presents comparison of patients with successful maintenance of SR and controls. Two patients of the control group developed AF during the follow-up period, and these patients were excluded from the comparison data.

The characteristics of patients who underwent electrical cardioversion or PVI were compared in Table 4. Both groups had similar age, sex distribution, and height. Patients in the electrical cardioversion group had higher bodyweight. No difference in hemodynamic parameters was seen. MPO (84.3 vs. 40.5 ng/l, *p* = 0.007) and NT-proBNP (991.0 vs. 115.5 pg/ml, *p* < 0.001) were higher in the cardioversion group. There were also more patients with persistent AF (74.1% vs. 20.8%, *p* < 0.001) and recurrence of AF (77.8% vs. 18.8%, *p* < 0.001) in the cardioversion group. No difference in left atrial (LA) parameters or antiarrhythmic drug use was seen.

Multivariable logistic regression analysis was performed for the study population with AF recurrence as a dependent variable. MPO (OR = 0.985, *p* = 0.010) was independently associated with AF recurrence when LA diameter, age, and AF type were included in the analysis (Table 5). Body mass index, pulse pressure, and systolic and diastolic BP were not associated with repeated episodes of AF (data not shown).

Interpreted predicted probabilities calculated for MPO are presented in Figure 3. For example, patients with MPO lower than 46 ng/ml at the baseline had at least a probability of 70% of maintaining SR after one-year follow-up period regardless of the selected intervention.

## 4. Discussion

The present study showed that patients with AF had higher levels of MPO, Gal-3, hsCRP, and NT-proBNP, compared to healthy controls, but there was no difference in oxLDL. Also, our secondary analysis showed that higher baseline MPO was independently associated with recurrent episodes of AF during the one-year follow-up period.

The pathogenesis of AF is complex and seems to be an interplay between inflammatory response [5, 6], OxS [7, 8], and development of atrial fibrosis [14]. These processes lead to the electrical and structural remodelling of the atria, which explains the progressive nature of the disease [14]. The prognostic role of different biomarkers in terms of the effectiveness of rhythm control therapies is an increasingly important focus in AF research. There is accumulating evidence that chronic inflammation can alter atrial electrophysiology, which may increase vulnerability to AF [5]. Several large prospective cohort studies like the Cardiovascular Health Study [15] have shown that CRP is associated with presence of AF and can also predict development of new-onset AF. Data also suggests that AF per se can uphold the inflammatory response in the organism, thereby contributing to atrial remodelling [1]. This causes a vicious circle that may contribute to the progressive nature of AF. Watanabe et al. [16] showed in their study that hsCRP was an independent predictor for both successful cardioversion of AF and its recurrence after electrical cardioversion. These results were also confirmed in a meta-analysis by Yo and colleagues [17]. Our study showed significantly higher hsCRP values for AF patients compared to the control group, which is consistent with previous studies. However, we did not find differences in the hsCRP baseline values between successful and unsuccessful maintenance of SR after one year. The reason for this might be the relatively short duration of AF before aggressive rhythm control was initiated and the symptomatic yet paroxysmal nature of AF in the patients with PVI. Also, we excluded patients with heart failure and other potential confounding factors, which might increase hsCRP levels. We did note lower baseline hsCRP levels in the control group versus SR maintenance group, suggesting a low-grade inflammatory response in all AF patients regardless of rhythm control outcomes.

Galectin-3 (Gal-3) is a protein of the lectin family that is involved in cell differentiation, fibrinogenesis, and inflammation [18]. Gal-3 seems to induce fibrosis by activating (myo)fibroblasts and endocardial cells through increasing the extracellular matrix (ECM) [19]. Evidence shows that Gal-3 is an important factor in the acute phase of inflammatory response, initiating neutrophil and mast cell activation, but is also involved in transition to chronic inflammation by causing fibrogenesis and tissue fibrosis [19]. Several studies have provided new insight into associations between Gal-3 and AF [20, 21]. Our study showed significantly higher Gal-3 levels in AF patients compared to controls. Moreover, we found statistically lower Gal-3 levels in the control group compared to the successful SR maintenance group, suggesting low-grade inflammatory and fibrotic processes in all AF patients. A recently published meta-analysis [22] considered Gal-3 as a predictor of AF ablation outcomes. The pooled findings showed higher levels of Gal-3 in patients with recurrent AF after ablation, and the association was independent of age, gender, and left atrial dimensions. The mean Gal-3 values in the analysis of the AF recurrence group ranged from 6.03 to 30.8 ng/ml and in the group with AF episodes from 5.7 to 24.5 ng/ml. Compared to the mean values for our study group (13.0 with AF recurrence vs. 11.7 ng/ml without AF recurrence), the values of Gal-3 were higher in most of the past studies. Also, based on literature research, most studies included a considerable proportion of patients with persistent AF, suggesting advanced stages of the disease. Considering maintenance of SR after one year, we did not detect a difference in Gal-3 between the AF groups. This might be due to the small sample size and the relatively early stages of the disease in our study group which is also supported by the low levels of Gal-3 in all of our AF patients.

B-type natriuretic peptide (BNP) and its nonactive form NT-proBNP are well known in the diagnosis of heart failure, yet their importance in AF is not so well established. The hormone is usually synthesized in response to increased wall stress in the heart that is mainly due to increased loading conditions. In AF patients, NT-proBNP reflects the volume overload in the atria but is also thought to be increased due to the high frequency of atrial contractions and local atrial inflammation [23]. NT-proBNP is also associated with fibrosis degree of the atria in patients with AF [24] and correlates with serum markers of collagen turnover [25]. Our study showed that patients with AF had higher NT-proBNP than controls. NT-proBNP was lower in the group that maintained SR during the follow-up period. Some population-based studies also suggest that NT-proBNP levels can predict new-onset AF irrespective of the other risk factors of AF [26]. Also, two meta-analyses have demonstrated the predictive role of NT-proBNP in assessing the recurrence rate of AF after ablation [27] and electrical cardioversion [28]. In the present study, NT-proBNP was not independently associated with AF recurrence when age, MPO, AF type, and LA diameter were used as variables. However, higher levels of NT-proBNP in the subgroup of patients with a more persistent form of AF were found. As NT-proBNP is a marker of volume overload in the atria [23] and seems to correlate with disease progression, then a strong relation between persistent AF and NT-proBNP could influence our analysis.

MPO plays an important role in the interaction between inflammation and OxS, leading to cardiac fibrosis [29]. MPO is an enzyme with bactericidal properties, which is mainly released by activated polymorphonuclear neutrophils [30]. Upon the activation of polymorphonuclear neutrophils, MPO is secreted into the extracellular environment of the tissue. There, MPO is oxidized and reacts with various molecules, which results in the generation of reactive oxygen species [30]. MPO causes the production of different hypohalous acids, most notably hypochlorous acid (HOCl), which has been shown to activate matrix metalloproteinases (MMPs) and to inactivate tissue inhibitors of MMP [29]. These processes among others lead to increased ECM turnover, collagen accumulation, and fibrosis in the atrial tissue [30]. MPO has been associated with various cardiovascular diseases [29], but the link to AF is not so well established. Only a few clinical studies have dealt with the role of MPO in association with AF. According to Li and colleagues [31], higher levels of MPO might be predictive of arrhythmia recurrence after AF ablation. A more recent study by Holzwirth et al. [32] including 23 patients with AF during PVI found elevated MPO levels compared to controls, but no differences in baseline MPO, irrespective of rhythm outcome. The authors hypothesized that this might have been due to the small sample size and the inclusion of a heterogeneous group of AF patients. Our findings showed higher levels of MPO in patients with AF and association with higher AF recurrence after electrical cardioversion or ablation (rhythm control) which is consistent with the study by Li and colleagues. Considering this, MPO might be a clinically valid prognostic marker for assessment of AF recurrence.

The role of nonphysiological OxS in development of AF is an increasingly studied topic. It has been found that, besides inflammation, nonphysiological OxS plays an important role in the atrial remodelling process [33]. Mihm et al. were the first to show a marked elevation of OxS markers in their studies with chronic AF patients undergoing Maze operation [34].

Several different markers of oxidative stress have been associated with AF [9], but information on the role of oxLDL is still limited. In a small study [35], oxLDL was higher in patients with AF without other risk factors and was associated with the development of hypertension. In the present study, we examined the importance of malondialdehyde-modified low-density lipoprotein (MDA-LDL), a subtype of oxLDL, which is a well-recognized risk marker for cardiovascular disease, mainly atherosclerosis [36]. We did not detect any difference in MDA-LDL levels between the study group and controls nor between patients with maintenance of SR and those with recurring AF. Also, Kimura et al. studied MDA-LDL levels in patients with AF undergoing PVI ablation, but they failed to see any difference between patients with AF recurrence and those with S maintenance after a median follow-up of 9.7 years [37]. But we found increased levels of MPO and Gal-3 in patients with AF, which are also substantial in the development of OxS [38, 39]. MPO targets apolipoprotein B-100, a unique protein of LDL, which causes formation of oxidized lipoproteins Mox-LDL [39]. These have been shown to trigger inflammation by activating endothelial cells and by inducing proinflammatory molecules like tumour necrosis factor *α* (TNF *α*) and interleukin 8 (IL-8) [39]. Gal-3 has been found to enhance the expression of lectin-like oxidized low-density lipoprotein (oxLDL) receptor-1 (LOX-1) in the endothelial cells. LOX-1 is the main receptor involved in the uptake of oxLDL thereby contributing to the endothelial dysfunction caused by oxLDL [40].

Our study failed to detect an increase in MDA-LDL in patients with AF. Because a clear increase in MPO and Gal-3 was observed, it can be argued that other markers of OxS, like Mox-LDL and LOX-1, might be more important in the early stages of AF and should be the focus of further studies on associations between OxS and AF.

The current study has some limitations to be addressed. The relatively small sample size might have limited the statistical power of the study. Also, as the patients were followed up periodically, there might have been some missed cases of asymptomatic clinical AF recurrence episodes. In addition to AF type and left atrial size, the used rhythm control strategy (PVI vs. cardioversion) is also expected to have an effect on sinus rhythm maintenance rate. Future prospective studies should address the predictive value of identified biomarkers for each AF subtype and for each treatment strategy.

## 5. Conclusions

Patients with AF had higher MPO, NT-proBNP, hsCRP, and Gal-3 levels compared to healthy controls. MPO and hsCRP were independently associated with AF. Lower baseline MPO levels were associated with better long-term outcomes after AF ablation or electrical cardioversion. These results indicate that inflammatory and fibrotic processes play an important role in the development of AF. MPO might be a clinically valid prognostic marker for assessment of AF recurrence after rhythm control therapy and needs further studies to confirm this hypothesis.

## Figures and Tables

**Figure 1:** Difference in markers of inflammation and fibrosis between AF patients and controls.

**Figure 2:** Difference in markers of inflammation and fibrosis between patients with successful and unsuccessful maintenance of SR during one-year follow-up.

**Figure 3:** Probability of successful maintenance of sinus rhythm compared to MPO levels.

**Table 1:** Demographic and clinical characteristics of AF patients and controls.

Variable	AF patients (*n* = 75)	Controls (*n* = 75)	*p* value
Age (years)	58 (±9)	57 (±11)	0.545
Male, *n* (%)	54 (72.0)	54 (72.0)	1.000
Height (cm)	175 (±10)	175 (±10)	0.949
Weight (kg)	90.1 (±16.6)	81.3 (±16.4)	0.001
Body mass index (kg/m^2^)	29.4 (±4.7)	26.4 (±3.7)	<0.001
Heart rate (beats per minute)	59 (±9)	61 (±8)	0.077
Peripheral systolic blood pressure (pSBP) (mmHg)	127 (±13)	128 (±15)	0.557
Peripheral diastolic blood pressure (pDPB) (mmHg)	79 (±9)	78 (±8)	0.861
Peripheral pulse pressure (pPP) (mmHg)	48 (±9)	50 (±11)	0.375
hsCRP (mg/l)	1.5 (0.9-3.8)	1.1 (0.6-2.0)	0.001
MPO (ng/l)	52.6 (31.9-86.0)	36.2 (20.9-54.9)	<0.001
Galectin-3 (mg/l)	11.4 (9.6-14.5)	9.7 (8.9-12.0)	0.003
oxLDL (U/l)	71.5 (60.5-94.3)	71.7 (56.3-87.7)	0.449
NT-proBNP (pg/ml)	209.0 (99.5-827.0)	28.0 (20.0-43.0)	<0.001
Ejection fraction (%)	58 (±9)	64 (±6)	0.015
Left atrial diameter (cm)	4.0 (±0.5)	3.6 (±0.4)	0.001
Left atrial end systolic volume index (ml/m^2^)	36.3 (±9.7)	23.3 (±4.5)	<0.001

Values are presented as mean ± SD or median (IQR) or count (%). SD: standard deviation; IQR: interquartile range; hsCRP: high-sensitivity C-reactive protein; MPO: myeloperoxidase; oxLDL: oxidized low-density lipoprotein; NT-proBNP: N-terminal pro-brain natriuretic peptide.

**Table 2:** Multivariable logistic regression analysis for diagnosis of atrial fibrillation.

Variables	OR (95% CI)	SE	*p* value
MPO	1.012 (1.004-1.024)	0.005	0.014
hsCRP	1.265 (1.041-1.579)	0.105	0.026
Weight	1.029 (1.006-1.053)	0.011	0.013

OR: odds ratio; CI: confidence interval; SE: standard error of logarithm of odds ratio; MPO: myeloperoxidase; hsCRP: high-sensitivity C-reactive protein.

**Table 3:** Demographic and clinical characteristics of AF patients with successful and unsuccessful maintenance of sinus rhythm after follow-up of one year and healthy controls.

Variable	Unsuccessful AF patients (*n* = 30)	Successful AF patients (*n* = 45)	Controls (*n* = 73)	*p* value (unsuccessful vs. successful)	*p* value (successful vs. controls)
Age (years)	59 (±10)	57 (±9)	57 (±11)	0.536	0.739
Male (%)	24 (80.0)	30 (66.3)	52 (71.2)	0.319	0.751
Height (cm)	175 (±11)	175 (±10)	175 (±10)	0.911	0.846
Weight (kg)	94.0 (±20.0)	87.6 (±13.6)	80.7 (±16.1)	0.102	0.018
Body mass index (kg/m^2^)	30.7 (±5.7)	28.6 (±3.6)	26.3 (±3.7)	0.055	0.001
Heart rate (beats per minute)	63 (±10)	56 (±8)	61 (±8)	0.002	0.001
Peripheral systolic blood pressure (pSBP) (mmHg)	124 (±14)	128 (±12)	128 (±16)	0.168	0.945
Peripheral diastolic blood pressure (pDPB) (mmHg)	78 (±8)	78 (±9)	78 (±8)	0.961	0.817
Peripheral pulse pressure (pPP) (mmHg)	46 (±8)	50 (±9)	50 (±11)	0.036	0.985
hsCRP (mg/l)	1.9 (1.0-4.4)	1.5 (1.2-3.1)	1.1 (0.6-2.0)	0.859	0.004
MPO (ng/l)	84.3 (42.9-132.5)	40.5 (31.0-71.7)	35.1 (20.8-55.4)	0.005	0.052
Galectin-3 (mg/l)	11.8 (10.9-14.4)	10.8 (9.3-14.5)	9.7 (8.9-12.0)	0.355	0.024
oxLDL (U/l)	67.2 (60.1-80.2)	75.7 (64.0-101.1)	71.7 (57.0-87.0)	0.107	0.165
NT-proBNP (pg/ml)	694.0 (241.0-1170.0)	127.5 (83.8-237.0)	28.0 (20.0-43.0)	<0.001	<0.001
Ejection fraction (%)	54 (±10)	61 (±8)	64 (±6)	<0.001	0.154
Left atrial diameter (cm)	4.0 (±0.5)	4.0 (±0.5)	3.6 (±0.4)	0.983	0.002
Left atrial end systolic volume index (ml/m^2^)	36.0 (±11.5)	36.6 (±8.4)	23.3 (±4.5)	0.797	<0.001

Values are presented as mean ± SD or median (IQR) or count (%). SD: standard deviation; IQR: interquartile range; hsCRP: high-sensitivity C-reactive protein; MPO: myeloperoxidase; oxLDL: oxidized low-density lipoprotein; NT-proBNP: N-terminal pro-brain natriuretic peptide.

**Table 4:** Demographic and clinical characteristics of AF patients who underwent electrical cardioversion or pulmonary vein isolation.

Variable	Electrical cardioversion (*n* = 27)	Pulmonary vein isolation (*n* = 48)	*p* value
Age (years)	59 (±10)	57 (±9)	0.370
Male, *n* (%)	20 (74.1)	34 (70.8)	0.974
Height (cm)	175 (±11)	175 (±10)	0.885
Weight (kg)	97.1 (±19.2)	86.2 (±13.6)	0.006
Body mass index (kg/m^2^)	31.8 (±6.0)	28.1 (±3.2)	<0.001
Heart rate (beats per minute)	63 (±10)	56 (±8)	0.002
Peripheral systolic blood pressure (pSBP) (mmHg)	124 (±15)	128 (±12)	0.271
Peripheral diastolic blood pressure (pDPB) (mmHg)	78 (±9)	79 (±9)	0.765
Peripheral pulse pressure (pPP) (mmHg)	46 (±9)	50 (±9)	0.154
hsCRP (mg/l)	2.3 (1.2-4.1)	1.5 (0.9-3.2)	0.223
MPO (ng/l)	84.3 (49.8-131.8)	40.5 (30.9-72.1)	0.007
Galectin-3 (mg/l)	11.4 (10.2-14.8)	11.1 (9.4-14.4)	0.613
oxLDL (U/l)	71.4 (61.9-89.2)	73.0 (59.6-94.2)	0.762
NT-proBNP (pg/ml)	991.0 (365.0-1240.0)	115.5 (81.0-231.0)	<0.001
Ejection fraction (%)	53 (±10)	61 (±7)	<0.001
Left atrial diameter (cm)	4.1 (±0.5)	4.0 (±0.5)	0.656
Left atrial end systolic volume index (ml/m^2^)	36.0 (±12.0)	36.5 (±8.3)	0.830
CHA2DS2-VASc score, *n* (SD)	1.8 (±1.2)	1.3 (±1.2)	0.070
AF type Paroxysmal, *n* (%) Persistent, *n* (%)	7 (25.9) 20 (74.1)	38 (79.2) 10 (20.8)	<0.001 <0.001
Antiarrhythmic drug None, *n* (%) Propafenone, *n* (%) Amiodarone, *n* (%) Flecainide, *n* (%)	5 (18.5) 17 (63.0) 5 (18.5) 0 (0)	5 (10.4) 27 (56.3) 8 (16.7) 8 (16.7)	0.524 0.747 0.909 0.064
Use of beta-blockers, *n* (%)	22 (81.5)	45 (93.8)	0.207
AF recurrence during 1-year follow-up, *n* (%)	21 (77.8)	9 (18.8)	<0.001

Values are presented as mean ± SD or median (IQR) or count (%). SD: standard deviation; IQR: interquartile range; hsCRP: high-sensitivity C-reactive protein; MPO: myeloperoxidase; oxLDL: oxidized low-density lipoprotein; NT-proBNP: N-terminal pro-brain natriuretic peptide.

**Table 5:** Multivariable logistic regression analysis for recurrence of atrial fibrillation.

Variables	OR (95% CI)	SE	*p* value
Age	1.014 (0.930-1.109)	0.044	0.757
LA diameter	0.767 (0.156-3.794)	0.798	0.740
AF type: persistent	0.016 (0.002-0.074)	0.886	<0.001
MPO	0.985 (0.970-0.994)	0.006	0.010

OR: odds ratio; CI: confidence interval; SE: standard error of logarithm of odds ratio; MPO: myeloperoxidase; AF type: paroxysmal or persistent atrial fibrillation.

## Data Availability

The data used to support the findings of this study are available from the corresponding author upon request.
